# Segmentation of Overlapping Cervical Cells with Mask Region Convolutional Neural Network

**DOI:** 10.1155/2021/3890988

**Published:** 2021-10-04

**Authors:** Jiajia Chen, Baocan Zhang

**Affiliations:** ^1^Zhongshan Hospital Xiamen University, Xiamen, Fujian 361004, China; ^2^Chengyi University College, Jimei University, Xiamen, Fujian 361021, China

## Abstract

The task of segmenting cytoplasm in cytology images is one of the most challenging tasks in cervix cytological analysis due to the presence of fuzzy and highly overlapping cells. Deep learning-based diagnostic technology has proven to be effective in segmenting complex medical images. We present a two-stage framework based on Mask RCNN to automatically segment overlapping cells. In stage one, candidate cytoplasm bounding boxes are proposed. In stage two, pixel-to-pixel alignment is used to refine the boundary and category classification is also presented. The performance of the proposed method is evaluated on publicly available datasets from ISBI 2014 and 2015. The experimental results demonstrate that our method outperforms other state-of-the-art approaches with DSC 0.92 and FPRp 0.0008 at the DSC threshold of 0.8. Those results indicate that our Mask RCNN-based segmentation method could be effective in cytological analysis.

## 1. Introduction

Cervical cancer is one of the most common types of cancer among women, which causes tens of thousands of deaths every year. In recent years, cytology test, such as Pap smear, is widely used to diagnose cervical cancer in its early precancerous stages. The successful detection of precancerous lesions is essential for effective treatment of the cancer [1]. Conventionally, the slides containing the cells from uterine cervix are stained and examined under a microscope by a cytologist or pathologist, to detect nucleus and cytoplasmic atypia. However, the sensitivity of the test is mainly affected by many factors, such as the overlap among the cells and smearing (e.g., the presence of mucus, blood, and inflammatory cells) [2]. Although the impact could be reduced by newer preparation techniques (such as ThinPrep), these factors would lead to a large variation in false-negative rate [3]. On the other hand, the diagnostic procedure requires a large amount of time and is tedious. These issues have motivated the development of automated diagnostic techniques. Those techniques are largely based on the cell images acquired by a digital camera connected to a microscope. For cell images, automatically segmenting cervical cells from overlapped clumps is fundamental and remains a highly challenging task.

In previous studies, many approaches have been proposed for complete segmentation of overlapping cervical cells [4–6]. This increase was probably motivated by the first and second overlapping cervical cell segmentation challenges held in the International Symposium on Biomedical Imaging (ISBI) 2014 and 2015. During the conferences, two high-quality datasets containing the original cell images and their annotations were made publicly available. And those two datasets make the evaluation and comparison of different segmenting methods possible. Lu et al. [4] segmented overlapping cells by joint optimization of multiple set functions, where each function had both intracell and intercell constraints. Phoulady et al. [6] proposed a framework to detect nuclei and cytoplasm in cervical cytology extended depth of field (EDF) images. The boundaries were first approximated by a defined similarity metric and refined in two steps by reducing concavity. The framework was also evaluated on the two public datasets mentioned above. Tareef et al. [7] introduced a multipass fast watershed-based method to segment both nucleus and cytoplasm from large cell masses of overlapping cells. They located the nuclei with barrier-based watershed and then segmented the isolated, partially overlapping cells with a watershed transform. At last, they proposed mutual iterative watersheds applied to each nucleus to estimate the cell shape. Liu et al. [8] proposed a morphological scaling-based topology filter. And they combined the topology filter with a newly derived mathematical toolbox into a multifunctional filtering algorithm 2D codimension two-object level set method, to split overlapping cells. The performance was evaluated quantitatively and qualitatively on the ISBI 2014 dataset.

Recently, deep learning has proven to be very successful in image classification, object detection, and instance segmenting. In deep learning, the convolutional neural network (CNN) is the most commonly used architecture for image analyzing tasks. The CNN models extract the underlying features of images automatically and do not need any a priori knowledge. For example, Moeskops et al. [9] proposed an automatic segmentation of MR brain images with a CNN. Additionally, the technique of transfer learning was exploited to overcome the lack of sufficient training data. Zhang et al. performed cross-subject seizure detection in EEGs using transfer learning [10].

Many CNN-based methods for cell segmentation have been proposed and published. Song et al. [11] presented a multiscale CNN to classify every pixel into the category of cytoplasm or background, where the accurate detection of nuclei was critical. The labeling results were fed into the dynamic multitemplate deformation model for boundary refinement. They also incorporated high-level shape information to guide segmentation. Tareef et al. [12] presented a segmentation framework on superpixelwise convolutional neural network and utilized a learning shape prior to delineate the contour of each individual cytoplasm. The shape prior was dynamically determined during the training process. Wan et al. [13] adopted TernausNet to classify the image pixels into nucleus, cytoplasm, or background. Then, a modified DeepLab (V2) model was used to perform cytoplasm segmentation. It was worthy of note that a synthetic method was used to generate cell masses containing overlapping cells in the paper. Although the experimental results on real or synthetic datasets demonstrated promising results, these deep learning-based methods were somehow complicated or required prior knowledge about the shape of cells. This motivated our work to develop a fully automatic cell segmentation model for highly overlapping cells.

In this paper, we present a new segmentation method for segmenting cell clumps using mask region convolutional neural network (Mask RCNN). The workflow of the method is depicted in Figure 1. The real and synthetic cytology images from ISBI 2014 and ISBI 2015 are used as the original datasets. Similar to many previous works using deep learning to perform cytoplasm segmentation, the original images are augmented by flipping and rotating. Then, the original images and augmented ones are divided into training, validating, and testing datasets for the subsequent Mask RCNN. Mask RCNN is basically an extension of Faster RCNN [14], by adding a branch for predicting object masks. In other words, Mask RCNN has three output branches (i.e., mask branch, bounding box branch, and category branch). Mask RCNN is a typical two-stage method. In stage I, feature maps from images are extracted by the backbone network. These feature maps are passed through a regional proposal network to return the candidate bounding boxes of instance objects. In stage II, RoI (Region of Interest) pooling layer brings these candidate bounding boxes to the same size. And then, the proposals are passed to fully connected layers to output the bounding boxes, masks of objects, and category.

In summary, the main contributions of this work include the following:

- A new method using Mask RCNN is proposed for segmentation of overlapping cervical cells, where small amount of annotated images is needed and any a priori knowledge about cells is not required
- Our proposed method achieves superior results compared to other state-of-the-art methods in some terms of measures

The rest of this paper is organized as follows.  Section 2 describes the method.  Section 3 gives the structure of the convolutional network and the detailed information of datasets.  Section 4 describes the experimental results and comparison with state-of-the-art results. The discussion is presented in Section 5.

## 2. Method

Each cell image contains many cells, where cells sometimes overlap at a high ratio. Because of the relative small size and high contrast with background of the nuclei, segmenting nuclei is generally easier than segmenting cytoplasm. In previous works, many methods have been proposed to segment nuclei. Phoulady et al. [6] used the geometric features that nuclei were represented by small uniform intensity dark and convex regions. Wan et al. [13] used TernausNet to assign each pixel to three labels (nucleus, cytoplasm, and background). Based on the locations of detected nuclei, the corresponding regions were used in the following task of cytoplasm segmentation. On the other hand, nucleus detection inaccuracies directly affect the outcome of final cytoplasm segmentation.

In this paper, a new method based on Mask RCNN is proposed for cytoplasm segmentation directly, without the detection of nuclei in the first place. The architecture of Mask RCNN is depicted in Figure 2. In detail, the ResNet50 is used as the backbone network, with weights pretrained on the famous dataset ImageNet. Mask RCNN has two stages. In stage I, Faster RCNN proposes candidate object bounding boxes. Then, those candidate bounding boxes are classified into two categories (background and foreground). Regression is used to refine the foreground bounding boxes, with respect to the ground truth annotations and anchor boxes. The dimension of feature maps is 7 × 7 in our experiments. RoI alignment uses bilinear interpolation to compute the exact values of the input features in each RoI bin. After RoI alignment, the features are passed to three branches. In stage II, the category and bounding box branches are the same as those of Faster RCNN. The 7 × 7 features are upsampled to 14 × 14 and then fed into the mask branch. For each RoI, the mask branch outputs a mask of size 28 × 28. The loss function of Faster RCNN is defined as follows [15]:

(1) $$\begin{array}{c} L\left(p_{i},t_{i}\right)=\frac{1}{N_{\text{cls}}}\underset{i}{\sum }L_{\text{cls}}\left(p_{i},p_{i}^{*}\right)+\frac{\lambda }{N_{\text{reg}}}\underset{i}{\sum }p_{i}^{*}L_{\text{reg}}\left(t_{i},t_{i}^{*}\right), \end{array}$$

where *p*_*i*_ is the probability of the *i*-th bounding box being foreground; *p*_*i*_^∗^ = 1 when the *i*-th bounding box is positive and zero otherwise; *t*_*i*_, *t*_*i*_^∗^ is the *i*-th bounding box's and corresponding ground truth box's parameterize coordinates, respectively; *N*_cls_ is the batch size; *N*_reg_ is the number of anchors. *L*_reg_ is the smooth *L*1 function defined as

(2) $$\begin{array}{c} \text{Smoot}{\text{h}}_{L1}\left(x\right)=\left\{\begin{array}{cc} 0.5x^{2}, & \left|x\right|<1,\\ \left|x\right|-0.5, & \text{otherwise}. \end{array}\right. \end{array}$$

*L*_cls_ is the two category log loss function defined as

(3) $$\begin{array}{c} L_{\text{cls}}=-\log\left[p_{i}p_{i}^{*}+\left(1-p_{i}\right)\left(1-p_{i}^{*}\right)\right]. \end{array}$$

The loss function of the mask branch, denoted by *L*_mask_, is defined as the average binary cross-entropy loss. For a RoI associated with ground truth class *k*, *L*_mask_ is only defined on the *k*-th mask. The total loss function is the sum of all three branches, defined as *L* = *L*_cls_ + *L*_box_ + *L*_mask_. For more detailed information about Mask RCNN, please refer to the original paper proposed by He et al. [15]. As an example, Figure 3 presents a cervical cytology image from ISBI 2014 with the ground truth cytoplasm annotations and the segmentation proposed by our method.

## 3. Datasets and Experimental Design

In 2014 and 2015, the first and second Overlapping Cervical Cytology Image Segmentation Challenges (ISBI 2014 and ISBI 2015 [4]) were held. During the conferences, two datasets of high-quality cervical cytology image and their ground truth cell segmentation were made publicly available. Those two challenges have greatly motivated the research about segmentation of overlapping cells. The first dataset (from ISBI 2014) consists of 135 synthetic and 8 real cervical cytology EDF images in the training set and 810 synthetic and 8 real cervical cytology EDF images in the test set. The synthetic images are created by minor transformation of background and brightness of different isolated cells in real EDF images. It should be noticed that the real EDF images in this dataset were released without annotations of individual cytoplasm. So those images were not used in our paper. The second dataset (from ISBI 2015) contains 8 real cervical cytology EDF images in the training set and 9 real ones in the test set, with both ground truth annotations of cytoplasm. As for the main difference of those two datasets, images from ISBI 2014 are of size 512 × 512 with 2-10 cells in each image, and images from ISBI 2015 are of size 1024 × 1024 with more than 40 cells in each image.

Table 1 describes the training and testing datasets used in our experiments. The training dataset consists of 900 synthetic images from ISBI 2014 and 8 real EDF images from ISBI 2015. The testing dataset contains 45 images from ISBI 2014 and 9 images from ISBI 2015.

In order to compare with the segmentation results proposed by other researchers on the same datasets, we adopt four widely used evaluation metrics. The dice similarity coefficient (DSC) of two regions *A* and *B* is defined as DSC = 2|*A*∩*B*|/|*A*| + |*B*|. A cell in ground truth is considered to be well segmented if a segmentation in the detection has DSC above a specific threshold with it. In our evaluation, we adopt the following values of DSC threshold: {0.5, 0.6, 0.7, and 0.8}. The object-based false-negative rate (FNRo) is defined as the rate of cells having a DSC below the threshold. At pixel level, true positive rate (TPRp) and false positive rate (FPRp) are also reported. Their definitions are as follows: TPRp = TP/(TP + FN), FPRp = FP/(FP + TN). Higher value of TPRp along with lower value of FPRp means better cell segmentation. During evaluation, a cell in ground truth is not counted in the metrics of TPRp and FPRp if there is no region in the segmentation result that has a DSC greater than the specific threshold.

In the training process, the pretrained weights on ImageNet for the backbone network ResNet50 are used. The cell images from ISBI 2015 of size 1024 × 1024 are resized using crop. And the size of batch normalization is 8 images per batch. The nonmaximum suppression thresholds are set to be 0.9 and 0.7 during training and testing, respectively. The test platform is a desktop system with Nvidia RTX 2080Ti and 128 GB memory running Debian.

## 4. Results and Comparison

We first report the qualitative results on both datasets by several examples. And then, quantitatively the performance of our method is evaluated in comparison with that of state-of-the-art approaches.

The final segmentation results on some cell images from datasets ISBI 2014 and ISBI 2015 are presented in Figure 4. Compared with synthetic cervical cell images (Figure 4(a)), the real cytology images (Figure 4(b)) contain much more cells with high overlapping ratio. Higher overlapping ratio makes the segmentation more difficult.

The segmentation performance is evaluated by four evaluation metrics (i.e., DSC, FNRo, TPRp, and FNRp), which are the original metrics in the two ISBI competitions. The quantitative results are listed in Table 2. As shown by the table, the mean DSC on dataset ISBI 2015 is a litter lower than that on dataset ISBI 2014, and the mean FNRo on dataset ISBI 2015 is a little higher than that on dataset ISBI 2014. Those results are likely to be caused by the fact that the cervical cell images from ISBI 2015 have much more cells with higher overlapping ratio than the cell images from ISBI 2014.

The dataset from ISBI 2014 provides not only the ground truth cell segmentation but also the number of cervical cells and the mean overlapping ratio between every pair of cells in synthetic images. Based on this information, we conduct additional experiments to evaluate the segmentation performance over cell images with varied number of cells and overlapping ratio. The overlapping ratio indicates the degree of coincide between two cells in the cell images. The metrics of DSC, TPR, and FNRo are used in the evaluation.  Figure 5 shows a graphical visualization of segmentation results in terms of the three metrics. As seen from those figures, our model can successfully segment cells from clumps with a small number of cells and high overlapping ratio. It can also effectively segment cells from clumps with a large number of cells (about 10 cells) and low overlapping ratio. In Figure 4(a), three typical segmentations of synthetic cell images are presented with automated detection. Figure 4(b) shows three real EDF cervical cytology images with automated segmentation.

Due to the fact that manual annotations of cell segmentation are tedious and very time-consuming, the number of real cytological images with ground truth segmentation is small. Synthetic images are relatively easy to generate from isolated cells in real EDF images. On the other hand, the training of deep neural network needs a large amount of samples with ground truth annotations. Therefore, in our experiments, the training dataset contains much more synthetic cytology images than real ones.

For comparison, we employ the same DSC threshold of 0.7. The experimental results are listed in Tables 3 and 4.

According to Table 3, our proposed method achieves the best performance in terms of FPRp and FNRo over the other methods. In particular, the object-based false-negative rate is much lower than that of the other methods. Our method obtains a comparable DSC (0.92), with about 2.2% improvement over the average value (0.9).

By examining the results in Table 4, our method achieves better results than other approaches in some metrics and slightly worse results in other metrics. In detail, our model achieves the second best and third best results in terms of DSC and TPRp, respectively. In terms of FPRp, our method achieves the best result by a little margin. However, when the DSC threshold is set to be 0.8, our proposed method shows a promising performance in cytoplasm segmentation. The results are presented in Table 5. Our proposed Mask RCNN model achieves the best results in terms of DSC and FPRp over other two methods. Specifically, our obtained DSC is 0.92 and FPRp is 0.0008.

Compared with results obtained by Wan et al. [13], our achieved TPRp is 0.94, with up to 4% improvement, but the metric of FNRo is a little higher. Our obtained FNRo is much lower than that achieved by Tareef et al. [7]. Those experimental results indicate that our proposed method can be used to effectively segment individual cytoplasm from cell clusters in real cytology images.

The python code is run on a PC with a powerful GPU Nvidia GTX2080Ti. It would take around 1.5 s for the algorithm to segment the overlapping cells in a real EDF image. But it should be noticed that the time for segmenting depends largely on hardware and code optimization.

## 5. Discussion

Segmenting cytoplasm in cytology images is one of the most challenging tasks in cervix cytological analysis. This situation is caused by many reasons. For example, cells in images overlap at a relatively high ratio. And the presence of mucus and blood makes the images fuzzy. It is a very challenging task to precisely annotate the boundary of every single cell in images. Therefore, automated segmentation based on computer technology is much needed.

In this work, the proposed method based on Mask RCNN produces robust results on the problem of segmenting cytoplasm from cell images with high overlapping ratio. The qualitative results shown in Figure 4 allow us to conclude that our method produces robust boundaries on synthetic and real cytology images. However, some cytoplasm embedded in clumps is not segmented well enough, especially in the real EDF images. Quantitatively, our proposed method achieves the best results in terms of DSC and FPRp over other state-of-the-art approaches at the DSC threshold of 0.8. However, compared with other approaches, our method achieves better results in some terms and worse results in other terms, at the same DSC threshold of 0.7 (as suggested by the Overlapping Cervical Cytology Image Segmentation Challenges in 2015). The percentage of correctly segmented cells is a little bit low when segmenting cells embedded in clumps with a large number of cells. As can be concluded from the experimental results (Table 2), the average FNRo is 0.04 and 0.24 over dataset ISBI 2014 and ISBI 2015, respectively. To the best of our knowledge, no published approaches have achieved superior performance in all four metric terms on the same test dataset.

Overall, the qualitative and quantitative evaluation demonstrates the efficiency of our proposed method for cell segmentation in cytology images. Compared with other approaches, our method does not need any prior knowledge of the shape of cells and could segment cytoplasm without any information of the nuclei. For instance, the level set-based segmentation methods require a number of arbitrary parameters empirically set of every dataset, such as in [12, 17, 18]. Some methods are based on shape deformation and detection, such as in [12]. Although shape-based method is one of reliable techniques for cell segmentation, it may lack strong generalization ability for insufficient cell shapes in the training dataset.

However, our method requires a large number of annotated cell images for training. On the other hand, our model tends to annotate small isolated clumps as cytoplasm, where those clumps of small area may be mucus or blood. One possible improvement is to utilize the information of shape and area of the cells. In the future work, we will modify our proposed model by filtering out candidate bounding boxes that have relatively small area. In addition, we will try to build a framework to further improve accuracy and efficiency. To our knowledge, the new CNN model BlendMask can effectively predict dense per-pixel position-sensitive instance features with few channels and learn attention maps for each instance with merely one convolution layer [19]. It has showed remarkable performance on some open datasets. A new model based on BlendMask could be our candidate method for segmentation of overlapping cervical cells.

## 6. Conclusion

In this paper, we present a Mask RCNN-based method that addresses the challenging task of segmenting cells in cytology images. The method requires neither prior knowledge of the shape of cells nor the detection of nuclei. Therefore, our method has relatively strong generalization ability. The experimental results on publicly available datasets show that our method achieves the best DSC of 0.92 and FPRp of 0.0008 at the DSC threshold of 0.8.

## Figures and Tables

**Figure 1:** Workflow of the segmentation for overlapping cell images using Mask RCNN.

**Figure 2:** The architecture of mask region convolutional neural network.

**Figure 3:** Example of segmentation of a cytology image: (a) the original overlapping cell image; (b) the ground truth segmentation; (c) the proposed segmentation using Mask RCNN.

**Figure 4:** Segmentation results on (a) synthetic cervical cell images from ISBI 2014 and (b) real cervical cell images from ISBI 2015.

**Figure 5:** The graphical visualization of segmentation results, by using the overlapping ratios and the different numbers of cells. The visualization over (a) DSC, (b) TPR, and (c) FNRo.

**Table 1:** The number of cell images in the datasets.

	Total	ISBI 2014	ISBI 2015
Training set	908	900	8
Testing set 1	45	45	
Testing set 2	9		9

**Table 2:** Segmentation performance with four evaluation metrics.

Dataset	Thresholding	DSC	TPRp	FPRp	FNRo
ISBI 2014	DSC > 0.5	0.92 ± 0.037	0.89 ± 0.057	0.001 ± 0.026	0.0056 ± 0.026
	DSC > 0.6	0.93 ± 0.032	0.89 ± 0.053	0.001 ± 0.0007	0.013 ± 0.054
	DSC > 0.7	0.93 ± 0.029	0.90 ± 0.048	0.001 ± 0.0007	0.022 ± 0.066
	DSC > 0.8	0.94 ± 0.022	0.91 ± 0.037	0.001 ± 0.0006	0.058 ± 0.127

ISBI 2015	DSC > 0.5	0.84 ± 0.032	0.90 ± 0.046	0.001 ± 0.0004	0.120 ± 0.067
	DSC > 0.6	0.87 ± 0.025	0.91 ± 0.049	0.001 ± 0.0003	0.200 ± 0.091
	DSC > 0.7	0.89 ± 0.022	0.92 ± 0.051	0.001 ± 0.0002	0.277 ± 0.093
	DSC > 0.8	0.92 ± 0.01	0.94 ± 0.029	0.0008 ± 0.0001	0.387 ± 0.131

**Table 3:** Comparison of segmentation performance on ISBI 2014 test dataset using DSC, TPRp, FPRp, and FNRo (DSC threshold = 0.7). The values are in the format of *μ* ± *σ*.

Method	DSC	TPRp	FPRp	FNRo
Tareef et al. [7]	0.89 ± 0.07	0.94 ± 0.07	0.005 ± 0.005	0.22 ± 0.24
Lee and Kim [16]	0.90 ± 0.08	0.88 ± 0.10	0.002 ± 0.002	0.14 ± 0.19
Lu et al. [4]	0.88 ± NA	0.92 ± NA	0.002 ± NA	0.21 ± NA
Wan et al. [13]	0.93 ± 0.04	0.93 ± 0.05	0.001 ± 0.002	0.11 ± 0.13
Liu et al. [8]	0.90 ± 0.07	0.91 ± 0.08	0.003 ± 0.005	0.28 ± 0.23
Our Mask RCNN	0.92 ± 0.02	0.90 ± 0.05	0.001 ± 0.0007	0.02 ± 0.06

**Table 4:** Comparison of segmentation performance on ISBI 2015 test dataset using DSC, TPRp, FPRp, and FNRo (DSC threshold = 0.7). The values are in the format of *μ* ± *σ*.

Method	DSC	TPRp	FPRp	FNRo
Tareef et al. [7]	0.85 ± 0.07	0.95 ± 0.07	0.004 ± 0.004	0.11 ± 0.17
Song et al. [11]	0.89 ± NA	0.92 ± NA	0.002 ± NA	0.26 ± NA
Lee and Kim [16]	0.88 ± 0.09	0.88 ± 0.12	0.001 ± 0.001	0.43 ± 0.17
Phoulady et al. [6]	0.85 ± 0.08	0.94 ± 0.06	0.005 ± 0.005	0.16 ± 0.22
Wan et al. [13]	0.92 ± 0.05	0.91 ± 0.05	0.001 ± 0.003	0.13 ± 0.15
Our Mask RCNN	0.89 ± 0.02	0.92 ± 0.05	0.001 ± 0.0002	0.27 ± 0.09

**Table 5:** Comparison of segmentation performance on ISBI 2015 test dataset using DSC, TPRp, FPRp, and FNRo (DSC threshold = 0.8). The values are in the format of *μ* ± *σ*.

Method	DSC	TPRp	FPRp	FNRo
Tareef et al. [7]	0.89 ± NA	0.97 ± NA	0.002 ± NA	0.59 ± NA
Wan et al. [13]	0.91 ± 0.06	0.90 ± 0.05	0.001 ± 0.002	0.28 ± 0.24
Our Mask RCNN	0.92 ± 0.01	0.94 ± 0.02	0.0008 ± 0.0001	0.38 ± 0.13

## Data Availability

The datasets used in this paper were made publicly available in the first and second Overlapping Cervical Cytology Image Segmentation Challenges in 2014 and 2015.
